The article "Dracocephalum kotschyi Boiss. In Vitro Efficacy on Growth and Apoptosis Induction in Leishmania major Promastigotes" was published in 2022. Journal: Biomed Res Int.

# *Dracocephalum kotschyi* Boiss. *In Vitro* Efficacy on Growth and Apoptosis Induction in *Leishmania major* Promastigotes

**DOI:** 10.1155/2022/8109264

**Published:** 2022-10-14

**Authors:** Neda Kosari, Faham Khamesipour

**Affiliations:** Shahrekord Branch, Islamic Azad University, Shahrekord, Iran

## Abstract

*Dracocephalum kotschyi* Boiss. is a plant generally used in modern medicine to treat many human illnesses. It is also used to prevent tumor cell proliferation throughout the world. This study's objective was to evaluate this plant's in vitro efficacy on growth and apoptosis induction in *Leishmania major* promastigotes. To do this, the essential oil is extracted for the test following the collection and identification of *D. kotschyi*. The essential oil was analyzed using a GC-MS analyzer. Promastigotes of *L. major* were cultured in RPMI-1640 media, and the MTT assay and a flow cytometry analysis were carried out on promastigotes that had entered the log phase. To differentiate between viable, necrotic, and apoptotic treated or untreated promastigotes, the flow cytometry method of double staining with annexin V-FLUOS and propidium iodide (PI) was used. Given the results obtained, 11 phytochemicals were identified in the essential oil of this plant. Copaene (22.15%), methyl geranate (16.31%), geranial (13.78%), and carvone (11.34%) were the main substances. The essential oil of *D. kotschyi* inhibits the proliferation of *L. major* promastigotes at 921 *μ*g/mL, 252 *μ*g/mL, and 416 *μ*g/mL, respectively, after 24 h, 48 h, and 78 h. The cells were divided into four quadrates based on cell phases using the flow cytometry approach by double staining with annexin V-FLUOS and propidium iodide (PI): necrosis (Q1), late apoptosis (Q2), early apoptosis (Q3), and viable (Q4) quadrates. Overall, it is apparent that the different concentrations induced cell apoptosis in promastigotes. Observation under the light microscope at ×100 magnification showed that the different doses of *D. kotschyi* essential oil caused apparent alterations in the treated promastigotes. In this work, *D. kotschyi* essential oils induce programmed death on *L. major* promastigotes. This study opens many research perspectives, such as investigating the mechanisms of action and the production of a phytomedicine based on this plant.

## 1. Background

Biologically active natural substances, including medicinal plants, have been used for decades to prevent diseases and treat cellular disorders. According to Kinghorn et al., many pharmacologically effective medications have been produced from natural resources, such as medicinal herbs [1]. Numerous plants' therapeutic potential for treating diseases is still being studied. The prevalence of medicinal plants among people worldwide is rising due to their low risk of adverse effects, accessibility, and affordability [2].

*Dracocephalum kotschyi* Boiss. is a medicinal plant of the Labiatae family used in many countries. It is an aromatic plant that grows in Iran's high, mountainous regions [3–6]. In traditional medicine, several medicinal properties have been attributed to it. So this plant is used to treat congestion, stomach aches, headaches, and liver disease [7–9]. *Dracocephalum kotschyi* is a plant usually used in modern medicine to treat many human illnesses and prevent tumor cell proliferation worldwide [10–12]. *D. kotschyi* has some of biological and pharmacological activities that have been described, counting antibacterial [13], anti-inflammatory, and antifungal effects [14]. This plant also has antispasmodic, analgesic, antihyperlipidemic, and immunomodulatory activity [15]. The different biological properties of this plant are due to the bioactive chemical compounds of this plant. The essential oil of *D. kotschyi* contains flavonoids, which have antimicrobial characteristics, whereas *α*-terpineol and limonene have antinociceptive qualities [15]. The anticancer effects are brought on by methoxylated flavones such as luteolin, isokaempferid, apigenin, crisimaritin, penduletin, and xanthomicrol [16]. For example, some *in vitro* and *in vivo* studies have shown that apigenin induces cell apoptosis [17, 18]. Indeed, apoptosis is a programmed cell death process that involves cascades of events depending on energy and various morphological features [17]. Extrinsic (death receptor) and intrinsic (mitochondrial) pathways play a significant role in the induction of apoptosis. Apigenin is an effective agent for triggering apoptosis through the intrinsic or extrinsic pathway in human cancer cells. Apigenin treatment of the prostate cancer cell lines PC-3 and DU145 resulted in apoptosis via decreasing Bcl-2 and Bcl-xL proteins and increasing the active form of the Bax protein [19]. Through altering the amount of mitochondrial protein expression, apigenin can also cause cell apoptosis via upregulating the expression of the Bim protein and decreasing the expression of the Mcl-1 protein. To cause mitochondria-dependent cell apoptosis, this synergizes with the Bcl-2 inhibitor ABT-263 [20]. The antioxidant activity of the plant is probably caused by polyphenolic compounds such as flavonoids, chlorogenic acid, phenylpropanoids, caffeic acid, and caffeic acid [16].

Additionally, it was established that *D. kotschyi* had cytotoxic, antiproliferative, and apoptotic effects on cancer cells *in vitro* [15]. According to one research, the most beneficial fractions were CH2Cl2, luteolin, and essential oil (EO), which caused morphological changes in the cells. The biological properties of luteolin include antioxidant, anti-inflammatory, and anticancer activities. For *D. kotschyi*, the effect of flavonoids on tumor cell inhibition has been reported. This plant's flavonoids are considered the most effective chemicals [15].

Of all the studies on the biological properties of *D. kotschyi*, very few have evaluated the *in vitro* efficacy of this plant on the growth and apoptosis induction in *Leishmania major* promastigotes. A variety of protozoa from the genus *Leishmania* cause the vector-borne disease leishmaniasis. It is an emerging disease with high morbidity and mortality rates [21]. It has three primary forms: cutaneous, mucocutaneous, and visceral. Several drugs are used to treat this disease, but high toxicity levels have been established for these drugs [22, 23]. Pentavalent antimonials, amphotericin B, paromomycin, and pentamidine are the most frequently prescribed drugs for leishmaniasis. These medications have serious side effects, must be taken in high dosages for long periods, and must be administered parenterally [24]. It has also been established that drugs capable of initiating apoptosis of *Leishmania* promastigotes would be very effective in treating this parasitic disease [25]. The simplest model for screening is the promastigote since the parasites grow in cell-free media [21]. The inhibition of promastigote multiplication is assessed within three days, during which the control organism multiplies three to six times. Since promastigotes are not the desired parasites, some researchers like this screening method due to its simplicity [21]. The multiple therapeutic uses of *D. kotschyi* are of particular interest. In this regard, the current study has evaluated the *in vitro* efficacy of this plant on the growth and apoptosis induction in *L. major* promastigotes.

## 2. Materials and Methods

### 2.1. Plant Material and Preparation of Essential Oil

In October 2019, the plant utilized in this study was collected in Isfahan, Iran. Prof. Ghanadian verified it at the pharmacognosy department. The pharmacy school herbarium had a reference specimen (No. 1519). We had permission to collect *Dracocephalum kotschyi* from the Research and Ethics Committee of Islamic Azad University, Shahrekord Branch (date 2021/12/08, IR.IAU.SHK.REC.1400.061).

The plant parts were mechanically pulverized using an electric mixer after the aerial parts of the plants were dried in the lab at 16°C in the shade. The essential oils were obtained after three hours of hydrodistillation with a Clevenger apparatus. The oil was put into sealed vials, dissolved in hexane (Merck, Darmstadt, Germany), and dried on anhydrous sodium sulfate before being stored in the dark at 4-6°C.

### 2.2. Analysis Using Gas Chromatography-Mass Spectrometry (GC/MS)

The essential oil was analyzed using a GC with an Agilent 7890A coupled to a 5975C mass detector with a triple quadrupole electron ionization (EI) mass analyzer. An HP-5 GC capillary column (30 m × 0.25 mm; film thickness 0.25 *μ*m) was used to prepare the GC. The oven was preheated to 50°C and left there for two minutes. It was increased by 8°C/min to 250°C and then 250-330°C by 3°C/min for 58 min. At a 2 mL/min flow rate, helium served as the carrier gas. The injector and detector were both operated at a temperature of 280°C. Ion source temperature (230°C), mass range (50-700), and ionization voltage were the MS's parameters (70 Ev). MSD ChemStation was the operating system that was used. The chemicals were identified by comparing the mass spectra and retention times to data from the literature [21].

### 2.3. Culture of *L. major* Promastigotes (MRHO/IR/75/ER)

Promastigotes of the Iranian standard strain of *L. major* (MRHO/IR/75/ER) were purchased from the Pasteur Institute (Tehran, Iran). According to previous research, *L. major* promastigotes (MRHO/IR/75/ER) were grown in RPMI-1640 medium (without phenol red) at 25 ± 1°C in 25 mM HEPES (pH 7.2) and enhanced with 10% heat-inactivated FBS, antibiotics (100 *μ*g/mL streptomycin and 100 IU/mL penicillin), and L-glutamine (2 mM). Each vial's culture was checked every day for bacterial and fungal contamination. At 25 ± 1°C, the flasks were incubated. The following assays were then run-on promastigotes that had reached the log phase. Three times were done for each test [23].

### 2.4. MTT Assay

A 3-(4, 5-dimethylthiazol-2-yl)-2, 5-diphenyltetrazolium bromide (MTT) kit was employed to obtain the 50% inhibitory concentration (IC_50_). In order to do it, 5 mg of MTT powder in 1 mL of PBS sterile solution (5 mg/mL) was dissolved to prepare the MTT reagent. A 96-well microplate was used for the MTT assay (5 mg/mL, 20 *μ*L/well). After adding 2 × 10^5^ promastigotes/100 *μ*L/well, *D. kotschyi* essential oil in different increasing concentrations ranging from 125, 250, 500, 1000, and 2,000 *μ*L/mL was added to treat the parasites. The plates are incubated at 25 ± 1°C for 24, 48, and 72 h. Promastigote viability using the MTT assay was examined. Then, absorbance at a wavelength of 540 nm was measured using an ELISA reader device. The following formula was used to determine the percentage of cells that were exposed and unexposed in the samples [25, 26]:

(1) $$\begin{array}{c} \text{Viable promastigotes }\left(\%\right)=\frac{\left(A_{T}-A_{B}\right)}{\left(A_{C}-A_{B}\right)}\times 100, \end{array}$$

where *A*_*T*_ is the absorbance of the exposed promastigotes, *A*_*C*_ is the absorbance of the unexposed promastigotes 2,000,000, and *A*_*B*_ is the absorbance of the blank.

Final results were compared to positive controls (promastigotes treated with 20 *μ*L of amphotericin B 20 *μ*g/mL) and negative controls (promastigotes treated with 100 *μ*L of DMSO 1% without essential oil) to determine the IC50 (that inhibited half of the promastigotes growth). Observation of morphological changes in treated and untreated promastigotes with D. kotschyi essential oil.

### 2.5. Flow Cytometry Analysis

Using the flow cytometry technique, double staining with annexin V-FLUOS and propidium iodide (PI) allowed us to differentiate between promastigotes that had been treated with essential oil and were viable, necrotic, or apoptotic, as well as between those that had not. Annexin-V can differentiate between necrotic cells (PI-positive/upper left) and normal cells (both annexin-V and PI negative/lower left), apoptotic cells (only annexin-V positive as early apoptosis/lower right), and late apoptosis cells (both annexin-V and PI-positive/upper right) [27]. Promastigotes of essential oil that had been treated (2 × 10^6^ parasites/mL) and those that had not were centrifuged for ten minutes at 1400*g* after being twice washed with cold PBS solution following the manufacturer's instructions. Then, they were incubated in 100 *μ*L of annexin-V FLUOS with PI for 15 minutes at room temperature and in a dark area. A FACS Calibur flow cytometer (Becton Dickinson, USA) was used to analyze the samples after they had been examined. The percentage of positive cells for each sample was calculated [27].

### 2.6. Relevance of the Methodology

The methodology used in this study is consistent with current regulations and institutional guidelines and is replicable. All references used have been provided for ease of understanding.

### 2.7. Statistical Analysis

The *in vitro* antileishmanial activity's IC50 was calculated using a linear regression test and SPSS software version 19 (SPSS Inc., Chicago, IL, USA). The means and standard deviation were calculated using ANOVA. Tukey's multiple comparisons test was used to compare each experimental batch to the control batch at varied concentrations (ANOVA two-way). The tests were conducted at a 5% significance level.

## 3. Results

### 3.1. Extraction Yield of Essential Oils and GC/MS Analysis

The yield of the extraction was 1.1%. There were found to be eleven substances. They represent 91.5 percent of the oil. Copaene (22.15%), geranial (13.78%), methyl geranate (16.31%), and carvone (11.34%) were the main substances [28].

### 3.2. The Number of Live Promastigotes at Different Concentrations of Essential Oil

Table 1 shows the number of live promastigotes at different concentrations of *D. kotschyi* essential oil after 24 hours, 48 hours, and 72 hours of incubation. This data shows that the number of live promastigotes after 72 hours of incubation is higher than after 48 hours. It is inferred from this finding that the essential oil of *D. kotschyi* affected the promastigotes of *L. major.*

Figure 1 shows the number of live promastigotes (1 × 10^6^) as a function of different doses (dose-response) of essential oil. This figure shows that as the dose or concentration of essential oil increases, the number of living promastigotes in the reaction medium decreases. We deduce from this that there is a dose-response reaction to the number of living promastigotes.

### 3.3. Effect of *D. kotschyi* Essential Oil on the Cell Proliferation of *Leishmania major* Promastigotes

Cell viability was used to determine the percentage of growth inhibition (GI%) and the half-maximal inhibitory concentration (IC_50_) of essential oil of *D. kotschyi* on *L. major* promastigotes. Essential oils were tested at the following concentrations: 125, 250, 500, 1000, and 2000 *μ*g/mL.  Figure 2 shows the comparative effects the essential oil concentrations on *L. major* promastigotes after 24-h, 48-h, and 72-h exposure. After 24 to 72 hours of incubation, the number of viable parasites increased considerably in the negative control, indicating the absence of inhibition. The positive control showed parasite inhibition after 48 and 72 hours of incubation. For the essential oil of *D. kotschyi*, it was noted that the inhibitory activity was concentration-dependent. The highest inhibitory activity of the essential oil is observed at the concentration of 2000 *μ*g/mL, so the higher the concentration, the higher the activity.

The half inhibitory concentration (IC50) of the different concentrations (250, 500, 1000, and 2000 *μ*g/mL) of essential oil on *L. major* promastigotes is determined and reported in Table 2. The concentrations of *D. kotschyi* essential oil vary with time.

### 3.4. Flow Cytometry Was Used to Identify Phosphatidylserine at the Outer Membrane of Apoptotic Cells

The difference between necrosis and apoptosis was made using an annexin-V FLUOS staining kit, and the results were evaluated using the flow cytometry method.  Figure 3 provides further information. The flow cytometric tests with 2000 *μ*g/mL and 1000 *μ*g/mL of essential oil at 24 and 48 hours resulted in a two-dimensional plot of Annexin V-FITC against PI. The FSC/SSC plot to the untreated cells was used to establish the analysis border (control). By placing the most significant number of dots in the Q4 region of the control sample, the borders of the four quadrants (Q1-Q4) were established. Based on the cell phases, the cells were divided into four quadrates: necrosis (Q1), late apoptosis (Q2), early apoptosis (Q3), and viable (Q4) quadrates. Overall, it was found that the different concentrations induced cell apoptosis of promastigotes. Additionally, after 42 hours of incubation, the experimental group's percentage of promastigotes in the early and late stages of apoptosis changed with time.

Light microscopic observation under ×100 magnification showed that different doses of *D. kotschyi* essential oil cause apparent alterations in treated promastigotes, including cytoplasmic condensation, cell shrinkage, and immobility after 24 hours. In contrast, no visible changes were observed in the control group in cell morphology and promastigote multiplication.  Figure 4 shows the morphological alterations in exposed and unexposed promastigotes throughout time.

## 4. Discussion

The main objective of this study is to evaluate the *in vitro* efficacy of *Dracocephalum kotschyi* on growth and apoptosis induction in *Leishmania major* promastigotes.

The biological activity, including anticancer, antidiabetic, analgesic, and cardioprotective hepatoprotective, and food potential of medicinal plants are due to the strength of secondary metabolites contained within the plant and the diversity of these secondary metabolites [29–31]. This study investigated for the first time the phytochemical constituents of the essential oil of *D. kotschyi* by the gas chromatography-mass spectrometry (GC/MS) analysis technique. This work identified eleven (11) different chemical groups in the essential oil of *D. kotschyi.* Copaene (22.15 percent), methyl geranate (16.31 percent), geranial (13.78 percent), and carvone (13.78 percent) were the most common compounds (11.34 percent). Khamesipour et al. [25] made the same findings. Shakib et al. [28] discovered oxygenated sesquiterpenes, monoterpene hydrocarbons, sesquiterpene hydrocarbons, and oxygenated monoterpenes in the essential oils of *D. kotschyi*. Flavonoids such as calycopterin, xanthomicrol, apigenin 4'-O-*β*-d-glucopyranoside, isokaempferide, luteolin, luteolin 7-O-*β*-d-glucopyranoside, acetin 7-O-*β*-d-glucopyranoside, luteolin 3'-O-*β*-d-glucuronide, and apigenin were also identified according to the works of Zeng et al. [32]. These variations can be related to several parameters: the season of harvest, the method of collection, the method of extraction, the maturity of the plant, and the conditions of drying and grinding. The constituents of this plant are thought to be responsible for its biological characteristics. Flavonoids do, in fact, possess antibacterial properties [33]. The anticancer effects are carried on by methoxylated flavones such as apigenin, luteolin, isokaempferid, crisimaritin, penduletin, and xanthomicrol [16, 34]. The antioxidant activity of this plant's essential oil is usually related to phenolic components such as caffeic acid, chlorogenic acid, and phenylpropanoids [35].

The majority of drugs used to treat leishmaniasis now have several limitations, including high toxicity, challenging treatment schedules, and the development of resistance. New, safer, more potent, and economically feasible drugs are urgently required to treat leishmaniasis. Medicinal herbal products have been used to treat multiple human diseases for thousands of years. The *in vitro* efficacy of *D. kotschyi* on growth and apoptosis induction in *L. major* promastigotes was evaluated in this study.

The impact of *D. kotschyi* on the proliferation of *L. major* promastigotes analyzed using the MTT cell proliferation assay showed that promastigotes in the untreated control group continued to proliferate in a time-dependent manner (from 24 hours to 72 hours). Contrarily, within 24 hours after treatment with *D. kotschyi*, the number of promastigotes decreases sharply, and the decreased continued again for 72 hours. There was a significant difference in promastigote proliferation after 72 hours when comparing *D. kotschyi*-treated promastigotes with untreated promastigotes from the control group. These data suggest that the essential oil of *D. kotschyi* affects cell proliferation and induces apoptosis of target cells. Similar findings regarding the antiproliferative and apoptosis-inducing activities of curcumin on *L. major* were made in the study of Elamin et al. [21]. The latter investigated curcumin's effect on the cell cycle and showed a curcumin-dependent increase of S-phase cells that reached about 33% versus 14% in the control group after 16 hours of incubation.

This phenomenon was investigated to determine whether apoptosis is the cause of the cell death process brought on by *D. kotschyi*. Using flow cytometry after Annexin V/propidium iodide (PI) staining, different *D. kotschyi* were used to treat *L. major* promastigotes for 48 hours before they were stained and sorted. Four cell groupings could be seen in the data. Viable cells (Annexin V-/PI-) in bottom left; early apoptotic cells (Annexin V+/PI-) in bottom right; late apoptotic cells (Annexin V+/P+) in top right; and necrotic cells (Annexin V-/PI+) in top left (Figure 2). The proportion of early and late apoptosis corresponded to the proportion of apoptosis after determining the percentage of spontaneous apoptosis. Significantly, the essential oil of *D. kotschyi* increased the rate of apoptosis-induced mortality, and this effect was dose-dependent. The number of promastigotes that underwent apoptosis changed with a dose-response. These data could be explained by the fact that the essential oil of *D. kotschyi* acted on the target cells through cell signaling pathways related to cell apoptosis. In medulloblastoma cells, apoptosis caused by plant extracts would be accomplished through the mitochondrial pathway by downregulating Bcl-2, an antiapoptotic effector downstream of Shh signaling, according to Elamin et al. [21]. The programmed cell death (apoptosis) induced by *D. kotschyi* on *L. major* promastigotes could effectively eliminate the parasite, thus providing an alternative treatment to modern drugs. The same observations were made in Shaabani et al. [36]. They worked on human cancer cells. It was demonstrated through their study that the essential oil of *D. kotschyi* induced apoptosis in human glioblastoma U87 cells in a dose-response manner. Additionally, compared to the control group, there were significantly more cells in the sub-G1 phase. The findings show that *D. kotschyi* extracts cause cell apoptosis in U87 cells, in addition to measuring the proliferation of U87 cells and investigating the apoptotic effects of *D. kotschyi* on glioma cells. Based on cellular function, *D. kotschyi* extracts would have acted on ROS. Several studies have shown that ROS is essential in controlling a number of cellular functions, such as cell proliferation, inflammatory responses, and cell death [37, 38]. The fact that *D. kotschyi* extracts have been shown to increase ROS levels in cells over time significantly supports the theory that *D. kotschyi* causes cell death by causing oxidative stress and an accumulation of reactive oxygen species. Furthermore, it is known that many alterations occur during apoptosis in three essential steps, namely, cell membrane modifications, the cytoplasmic or mitochondrial pathway, and cell nucleus modifications [37, 38]. Different doses of *D. kotschyi* essential oil cause apparent alterations in treated promastigotes, such as cell shrinkage, cytoplasmic condensation, and immobility, beginning within 24 hours, according to light microscopic examination at a magnification of ×100.

This activity would be caused by the presence of luteolin, naringenin, penduletin, xanthomicrol, apigenin, isokaempferide, cirsimaritin, and calycopterin, according to Moghaddam et al. [39]. Cirsimaritin, penduletin, xanthomicrol, and calycopterin are methoxylated hydroxyflavones that were specifically effective against tumor cells. Luteolin caused tumor cells to undergo apoptosis, showing that it has apoptosis-inducing effects on the target organ [34]. Therefore, the main components of *D. kotschyi* and its isolated compounds exhibit a variety of activities affecting several targets and participate in the induction of apoptotic cell death in cancer, providing information on how to improve the effectiveness of cancer medications in people [34].

## 5. Conclusion

There are now new possibilities for treating leishmaniasis due to natural substances previously used in traditional medicine. On *L. major* promastigotes, the essential oil of *D. kotschyi* exerts lethal effects that cause the parasite to induce apoptosis. More research is required to understand further this natural substance's method of action and its toxic effects on other cells, particularly *in vitro*.

## Figures and Tables

**Figure 1:** Number of live promastigotes (1 × 10^6^) as a function of different doses (dose-response) of essential oil.

**Figure 2:** Comparison effects of the concentrations of the essential oil on *Leishmania major* promastigotes. ^∗∗^*p* < 0.01, ^∗∗∗^*p* < 0.001.

**Figure 3:** Differentiate between viable, necrotic, and apoptotic treated or untreated promastigotes with essential oil by flow cytometry analysis. Legends: (a) 2000 *μ*g/mL 24 h =50.7% (*Q*2 + *Q*3) induced cell apoptosis; (b) 1000 *μ*g/mL 24 h =25.24% (*Q*2 + *Q*3) induced cell apoptosis; (c) 2000 *μ*g/mL 48 h =86% (*Q*2 + *Q*3) induced cell apoptosis; and (d) 1000 *μ*g/mL 48 h =29.3% (*Q*2 + *Q*3) induced cell apoptosis.

**Figure 4:** Analysis of the morphology of *L. major* treated with *D. kotschyi* essential at 0, 24, 48, and 72 hours after treatment using light microscopy (magnification, × 100).

**Table 1:** The number of live promastigotes (1 × 10^6^) at different concentrations of essential oil and as a function time.

Concentration (*μ*g/mL)	24 h	48 h	72 h
125	0.85 ± 0.01	0.68 ± 0.01	0.69 ± 0.097
250	0.84 ± 0.011	0.61 ± 0.04	0.68 ± 0.03
500	0.82 ± 0.007	0.60 ± 0.07	0.660 ± 0.03
1,000	0.78 ± 0.014	0.58 ± 0.02	0.63 ± 0.08
2,000	0.72 ± 0.068	0.57 ± 0.05	0.58 ± 0.03
Positive control	0.74 ± 0.007	0.63 ± 0.04	0.68 ± 0.04
Negative control	0.86 ± 0.01	0.88 ± 0.04	0.99 ± 0.04

**Table 2:** IC_50_ at 24 hours, 48 hours, and 72 hours and *R*^2^.

Time	IC_50_ (*μ*g/mL)	*R* ^2^
24 hours	921	0.89
48 hours	252	0.84
72 hours	416	0.94
Positive control	255	0.87

## Data Availability

All data generated or analyzed during this study are included in this article. The datasets used and/or analyzed during the current study are also available from the corresponding author.
